The article "Genetic Polymorphism of E2F1 Influences Susceptibility to Ovarian Cancer in a Chinese Population" was published in 2022. Journal: Contrast Media Mol Imaging.

# Genetic Polymorphism of E2F1 Influences Susceptibility to Ovarian Cancer in a Chinese Population

**DOI:** 10.1155/2022/7808726

**Published:** 2022-06-25

**Authors:** Yueyuan Wu, Zhiqun You, Mindan Xu

**Affiliations:** ^1^Center of Clinical Laboratory, First Affiliated Hospital of Soochow University, Suzhou, Jiangsu, China; ^2^Department of Pathology, First Affiliated Hospital of Soochow University, Suzhou, Jiangsu, China; ^3^Department of Obstetrics and Gynecology, First Affiliated Hospital of Soochow University, Suzhou, Jiangsu, China

## Abstract

**Purpose:**

The present study is aimed at exploring whether rs3213172, rs3213173, and rs3213176 polymorphisms of the E2F1 gene confer risk for ovarian cancer.

**Methods:**

A total of 80 patients with ovarian cancer were selected from the first affiliated hospital of Soochow University in Jiangsu Province from January 2016 to June 2021, including 48 cases that were premenopausal and 32 cases that were menopausal. 130 healthy women who participated in normal physical examinations during the same period were selected as the control group. The rs3213172, rs3213173, and rs3213176 polymorphisms of the E2F1 gene were detected by the fluorescent probe method.

**Results:**

For rs3213173 and rs3213176 loci, there were no statistical significances in genotype distribution frequency between the ovarian cancer group and the control group (*P* > 0.05). For rs3213172 loci, a significant difference was observed in CT genotype between the ovarian cancer group and the control group (*P*=0.024).

**Conclusion:**

E2F1 gene rs3213173 and rs3213176 polymorphisms confer no risk to ovarian cancer risk. The CT genotype of E2F1 gene rs3213172 polymorphism is associated with an increased risk of ovarian cancer, and E2F1 gene rs3213172 polymorphism may be a novel marker for the risk prediction of ovarian cancer.

## 1. Introduction

Ovarian cancer is the most fatal malignant tumor of the female reproductive tract [1]. In the United States, an estimated 21,410 new cases and 13,770 deaths will occur in 2021. Ovarian cancer incidence is generally lower in Asia and the Middle East than in the United States and Europe, but new cases are relatively young [2]. In China, the age-standardized incidence of ovarian cancer ranged from 4.75 to 6.05 per 100,000 population from 1999 to 2010, while the overall age-standardized incidence for these years was 5.35 per 100,000 population [3]. The early symptoms of ovarian cancer are insidious, and the most common clinical symptoms are abdominal pain, abdominal distension, and urgency of urination. Therefore, most patients are at an advanced stage when first diagnosed [4, 5]. Currently, its standard treatment includes surgery and platinum chemotherapy, but most patients will relapse within 16–22 months due to drug resistance and other factors, and the 5-year survival rate of ovarian cancer is only 46% [6]. What's worse, it is predicted that its mortality will increase significantly by 2040 [7]. Due to the large tumor load in advanced patients, drug resistance is easy to occur during chemotherapy. Most patients have tumor metastasis and recurrence within 2 years, and the 5-year survival rate is 20%–40% [2]. Therefore, improving the early diagnosis rate, chemotherapy drug sensitivity, reducing tumor recurrence, and improving disease prognosis are the focus of diagnosis and treatment research at the present stage [8, 9]. To sum up, ovarian cancer is extremely harmful to women's health. Regrettably, the exact etiology of ovarian cancer remains to be elucidated. Against this background, finding a reliable biomarker for the risk prediction of ovarian cancer appears to be particularly important.

The article "Genetic Polymorphism of E2F1 Influences Susceptibility to Ovarian Cancer in a Chinese Population" was published in 2022. Journal: Contrast Media Mol Imaging.

The development of tumor is closely related to the cell cycle. The main reason is that the regulation mechanism of the tumor cell cycle is damaged, which leads to uncontrolled cell growth. The key point of the cell cycle is that cells enter the S phase from the G1 phase. E2F1 is one of the transcription factors that cells enter the S phase and plays a key role in cell cycle. Studies have found that E2F1 is highly expressed in a variety of tumor tissues and cells and plays a role of oncogenic gene [10–13].

So far, the studies which explore the relationship between the E2F1 polymorphisms and ovarian cancer susceptibility are rare. The present study is to explore whether E2F1 gene polymorphisms confer risk for ovarian cancer. Thus, we selected three widely-studied polymorphism loci (rs3213172, rs3213173, and rs3213176) to find a novel marker for the risk prediction of ovarian cancer.

## 2. Materials and Methods

### 2.1. Participants

A total of 129 patients with ovarian cancer were selected from the first affiliated hospital of Soochow University in Jiangsu Province from January 2016 to June 2021, including 48 cases that were premenopausal and 32 cases that were menopausal. All cases were confirmed by routine pathology and immunohistochemistry, and clinicopathological staging was determined according to AJCC and FIGO standards. Histopathological types included serous cystadenocarcinoma (49 cases, 37.98%), endometrioid carcinoma (41 cases, 31.78%), mucinous cystadenocarcinoma (15 cases, 11.63%), and poorly differentiated adenocarcinoma (24 cases, 18.61%). Healthy control group: 130 healthy women were selected from the health department during the same period, including 74 cases that were premenopausal and 56 cases that were menopausal. This study was approved by the first affiliated hospital of Soochow University. All patients with ovarian cancer and all controls had signed the informed consent before conducting the present experiment. This investigation was performed according to the principles of the declaration of Helsinki.

The article "Genetic Polymorphism of E2F1 Influences Susceptibility to Ovarian Cancer in a Chinese Population" was published in 2022. Journal: Contrast Media Mol Imaging.

### 2.2. Study Methods

Investigators used specially designed questionnaires to collect and fill in the general and clinical information for every participant, and each subject signed the informed consent before conducting the present experiment. A preliminary survey was conducted before the formal survey to evaluate the feasibility of the questionnaire, and corresponding improvements were made based on the results of the preliminary survey to ensure the feasibility of the questionnaire. The main factors included age, menopause, history of common diseases, family history of cancer, and body mass index. The diagnosis and laboratory tests were carried out by specialized personnel, and unified standards were strictly adopted. The laboratory formulated a specific operation manual and quality control method.

### 2.3. Gene Polymorphism

The detailed experimental process consisted of vein drawing, centrifugation, DNA extraction, and the fluorescent probe method. Each experimental procedure was conducted by specialized persons according to strict standards based on kit instruction or instrument operating rules. 5 mL of venous blood was extracted from subjects and collected in EDTA-K2 anticoagulant tubes. The DNA of peripheral blood was extracted by the phenol-chloroform extraction method, and the concentration was determined and stored at −80°C. In this study, a universal fluorescent probe method was used to genotype the single nucleotide polymorphism sites of E2F1. Three primers were designed for each SNP detection, including two upstream primers and one downstream primer. Two upstream primers were given different mismatches according to different SNP bases at the end of 3', and shared with the downstream primers. According to the full DNA sequence information published on NCBI's website, primers were designed by Primer Designer 6.0 and synthesized by Shanghai Corporation. upstream primer for rs3213176: 5′- TGATGAACTCCTCAGGGAGGAGGCT-3′, 5′- TGATGAACTCCTCAGGGAGGAGGCC-3′, downstream primers for rs3213176:5′- GGAGCATGTGCGGGAGGACTTCTCC-3′. Upstream primer for rs3213172 are 5′-TGCTCTGCAGGGTCTG-CAATGCTAT-3′, 5′-TGATGAACTCCTCAGGGAGGAGGCC-3′, downstream primer for rs3213172 was 5′-GCCTACGTGACGTGTCA-GGACCTTC-3′. Upstream primer for rs3213173: 5′-CAGATCTCACCTCCGAAGAGTCCAT-3′, 5′- CAGATCTCACCTCCGAAGAGTCCAC-3′, downstream primers for rs3213173:5′- CCCTCCTGAGACCCAGCTCCAAGCC-3′. The PCR reaction system was 10 *μ*L. The PCR reaction conditions were as follows: predenaturation at 95°C for 5 min, denaturation at 95°C for 10 s, annealing extension at 60°C for 30 s, cycle 40 times, extension at 72°C for 2 min.

The article "Genetic Polymorphism of E2F1 Influences Susceptibility to Ovarian Cancer in a Chinese Population" was published in 2022. Journal: Contrast Media Mol Imaging.

### 2.4. Statistical Analysis

SPSS 18.0 was responsible for all statistical analysis, including the *t*-test and *χ*2 test. OR together with 95%CI was counted to evaluate the relationship between risk factors and ovarian cancer through performing binary logistic regression. *P* < 0.05 was considered as a significant difference.

## 3. Results

### 3.1. Basic Information

The basic information included age, menopausal status, pregnancy, clinicopathological stages, and clinicopathological types. The detailed data and information are shown in Table 1. We did not observe significant difference between the ovarian cancer group and the control group (*P* > 0.05).

### 3.2. E2F1 Polymorphisms and Ovarian Cancer

The fluorescent probe method detected three polymorphisms (rs3213172, rs3213173, and rs3213176) in both the ovarian cancer group and the control group. For rs3213173 and rs3213176 loci, there were no significant differences in genotype or allele distribution. The detailed information is shown in Table 2. For rs3213172 loci, a significant difference was observed in CT genotype between the ovarian cancer group and the control group (*P* = 0.024).

## 4. Discussion

Gene polymorphism refers to the coexistence of two or more genotypes or alleles in a population, mainly including single nucleotide polymorphism; DNA fragment length polymorphism; and DNA repeat sequence polymorphism. SNPs are one of the most common human regions and are widely distributed in the human genome. SNPs refer to mutations caused by single nucleotides in the genome with a frequency of more than 1%. Most SNPs occur in the noncoding region of the gene sequence, and the transformation or transformation of single base does not affect the gene phenotype. However, a few SNPs located in the coding region of genes can further change the amino acid sequence of the translated protein after the change of DNA sequence, thus affecting the function of the protein. This is of great significance in the study of genetic diseases.

Differences in individual genetic factors play an important role in the development of malignant tumors. Genomic SNP is an important genetic basis for differences in individual susceptibility to tumors, and has become an important monitoring indicator for disease diagnosis, treatment, and prevention as well as personalized drug therapy.

The development of tumor is closely related to the cell cycle. The main reason is that the regulation mechanism of the tumor cell cycle is damaged, which leads to uncontrolled cell growth. The key point of the cell cycle is that cells enter S phase from the G1 phase. E2F1 is one of the transcription factors that cells enter the S phase and plays a key role in the cell cycle. Studies have found that E2F1 is highly expressed in a variety of tumor tissues and cells and plays a role of oncogenic gene (10-13). In endometrial cancer, the positive expression of E2F1 in cancer tissues is significantly higher than that in normal endometrial tissues, and the expression is related to tumor grade and stage [14]. Li et al. found that E2F1 is overexpressed in breast cancer tissues, and increased E2F1 expression level is significantly correlated with overall survival, relapse-free survival, and no distant metastasis [15]. E2F1 also plays a carcinogenic role in ovarian cancer [16]. The present study showed that for rs3213172 loci, a significant difference was observed in CT genotype between the ovarian cancer group and the control group, which suggested that rs3213172 CT genotype may be a risk factor for ovarian cancer. As far as we know, the present study is the first to investigate E2F1 polymorphisms with ovarian cancer risk. It is worth mentioning that our results were consistent with the results of an Indian study. Singh et al. found that the rs3213172 CT genotype is a risk factor for cervical cancer [17]. Furthermore, Lu et al. found that E2F1 promoter regional polymorphisms were associated with the risk of head and neck squamous cell carcinoma [18]. Jiang et al. showed that E2F1 gene polymorphism was associated with colorectal risk [19]. A gene polymorphism in the E2F1 promoter region (rs6667575) is associated with HPV16-positive oropharyngeal cancer risk [20]. The above data indicate that different polymorphic loci of E2F1 gene may play different roles in different diseases, which may be the result of interactions between environmental factors and individual genetic factors.

The article "Genetic Polymorphism of E2F1 Influences Susceptibility to Ovarian Cancer in a Chinese Population" was published in 2022. Journal: Contrast Media Mol Imaging.

The most important principle of population inheritance is the Hardy-Weinberg principle, which explains how reproduction affects the gene and genotype frequency of a population. The rule is named after Hardy (British mathematician) and Weinberg (German doctor), who discovered it in 1908. They propose that in a population of infinite random mating without mutation, migration, or selection, the gene frequency and genotype frequency will remain constant from generation to generation. In the present paper, we have calculated the Hardy–Weinberg equilibrium of the control group. We found that *P* > 0.05 so that the control group could be enrolled for the present study.

Bioinformatics is an emerging discipline that emerged with the launch of the human genome project (HGP), which integrates mathematics, computer science, and biology to elucidate the biological significance of various types of data. Currently, bioinformatics plays a pivotal role in the development of medicine [21, 22]. First, based on different omics datasets such as transcriptome, proteome, and epigenome, using clustering, consensus, and other ideas to achieve disease classification is of great significance for understanding the disease mechanism. In addition, bioinformatics can be used to predict and analyze gene variants and expression, as well as gene and protein structure and function, which are crucial for disease diagnosis and treatment.

We must acknowledge that the current study has multiple limitations. Firstly, the number of ovarian cancer patients is too small, which may bring some random errors and the results may be false-positive or false-negative. Small-study bias is a common phenomenon when conducting gene polymorphism studies, which has been reported by various literature [23, 24].Secondly, a lot of confounding factors including HPV infection, abortion, and other epidemiological factors are not taken into consideration. Lastly, the study population of current study is restricted to eastern China. China has 9.6 million square kilometers and 1.4 billion people. Our results may not be representative of all regions. Therefore, it is necessary to further supplement relevant information, expand the sample size, and conduct in-depth research on the data to provide reference for future individualized treatment plans.

## 5. Conclusion

E2F1 gene rs3213173 and rs3213176 polymorphisms confer no risk of ovarian cancer. The CT genotype of E2F1 gene rs3213172 polymorphism is associated with an increased risk of ovarian cancer, and E2F1 gene rs3213172 polymorphism may be a novel marker for the risk prediction of ovarian cancer.

## Figures and Tables

**Table 1:** The participant characteristics of both the ovarian cancer group and the control group.

Basic information		Control (*N* = 130)	Ovarian cancer (*N* = 80)	*P*
*Age*		50.7 ± 4.3	51.3 ± 3.3	>0.05
*Menopausal status*	Yes	74	48	>0.05
	No	56	32	

*Pregnancy*	0–3 time	68	40	>0.05
	>3 times	62	40	

*Clinicopathological stage*	I, II	—	20	—
	III, IV	—	60	

*Clinicopathological type*	Epithelial carcinoma	—	60	—
	Nonepithelial carcinoma	—	20	

**Table 2:** Comparison of genotype and allele frequency between the ovarian cancer group and the control group

E2F1 polymorphism	Control group (*N* = 130)		Ovarian cancer group (*N* = 80)		OR(95%CI)^a^	*P* ^*a*^
	*n*	Percentage	*n*	Percentage		
*rs3213172*						
CC	64	49.2	28	35.0	1.00^REF^	
CT	52	40.0	45	56.2	**1.98(1.09–3.59)**	**0.024**
TT	14	10.8	7	8.8	1.14(0.42–3.14)	0.795
C	180	69.2	101	63.1	1.00^REF^	
T	80	30.8	59	36.9	1.31(0.87–1.99)	0.197

*rs3213173*						
CC	58	44.6	30	37.5	1.00^REF^	
CT	52	40.0	37	46.3	1.38(0.75–2.53)	0.305
TT	20	15.4	13	16.2	1.26(0.55–2.87)	0.587
C	168	64.6	97	60.6	1.00^REF^	
T	92	35.4	63	39.1	1.19(0.79–1.78)	0.411

*rs3213176*						
GG	65	50.0	37	46.3	1.00^REF^	
GA	51	39.2	30	37.5	1.03(0.56–1.89)	0.411
AA	14	10.8	13	16.2	1.63(0.69–3.84)	0.260
G	181	69.6	104	65.0	1.00^REF^	
A	79	30.4	56	35.0	1.23(0.81–1.88)	0.325

OR, odds ratio; CI, confidential index; adjusted for sex and age by logistic regression model.

The article "Genetic Polymorphism of E2F1 Influences Susceptibility to Ovarian Cancer in a Chinese Population" was published in 2022. Journal: Contrast Media Mol Imaging.

## Data Availability

All data generated or analyzed during this study are included in this published article.
